# Comparative Efficacy of Routine Physical Therapy with and without Neuromobilization in the Treatment of Patients with Mild to Moderate Carpal Tunnel Syndrome

**DOI:** 10.1155/2022/2155765

**Published:** 2022-06-22

**Authors:** Muhammad Junaid Ijaz, Hossein Karimi, Ashfaq Ahmad, Syed Amer Gillani, Naveed Anwar, Muhammad Asad Chaudhary

**Affiliations:** ^1^University Institute of Physical Therapy, University of Lahore, Lahore, Pakistan; ^2^Nur International University, Lahore, Pakistan; ^3^Department of Biomedical Engineering, Kaohsiung Medical University, Taiwan

## Abstract

**Background:**

Median nerve mobilization is a relatively new technique that can be used to treat carpal tunnel syndrome. But literature about additional effects of neuromobilization for the management of carpal tunnel syndrome is scarce.

**Objective:**

To examine and compare the role of median nerve neuromobilization at the wrist as compared to routine physical therapy in improving pain numeric pain rating scale (NPRS), range of motion (Ballestero-Pérez et al., 2017), muscle strength, and functional status.

**Methods:**

A sample size of 66 patients was recruited using convenient sampling and distributed randomly in two groups. After assessing both groups using ROM, manual muscle strength, pain at NPRS, and functional status on the Boston Carpal Tunnel Syndrome Questionnaire (BCTQ), which consists of two further scales (the symptom severity scale (SSS) and the functional status scale (FSS)), Group 1 received conservative treatment including ultrasound therapy two days a week for six weeks, using a pulsed mode 0.8 W/cm^2^ and frequency 1 MHz, wrist splinting, and tendon gliding exercises, while Group 2 received both conservative treatments including ultrasound, splinting, and tendon gliding exercises as well as a neuromobilization technique. Treatment was given for 6 weeks, 2 sessions/week, and patients were reassessed at the end of the 3^rd^ and 6^th^ weeks.

**Results:**

Although both groups improved significantly in terms of all the outcome measures used, the neuromobilization groups showed a statistically more significant increase in flexion, extension, decrease in pain, decrease in SSS, decrease in FSS, and BCTQ as compared to the routine physical therapy group.

**Conclusions:**

The addition of neuromobilization in the rehabilitation program of carpal tunnel syndrome has better effects on treatment outcomes.

## 1. Introduction

Carpal tunnel syndrome (CTS) is a widespread compressive peripheral neuropathy that involves the entrapment of the median nerve in its passage at the carpal tunnel in the wrist [1, 2]. Padua et al. classify the severity of CTS based on electrophysiological findings into six categories: extreme CTS, severe CTS, moderate CTS, mild CTS, minimal CTS, and negative CTS. Using this neurophysiological classification, the CTS groups appeared normally distributed (extreme 3% of cases, severe 14%, moderate 36%, mild 24%, minimal 21%, and negative 3%) [3–5]. In the carpal tunnel, mechanical pressure applied to synovial tissue can result in biomechanical changes in the underlying tissues [6], which can thus elevate intracarpal pressure and increase symptoms [7, 8].

CTS patients indicate signs and symptoms of tingling, numbness, and night-time burning aches of the affected hand. Clinical signs may include a decreased fine motor skills and feeling light touch sensation. In severe cases, there is loss in grasping and squeezing strength of affected hand [9]. The causes of CTS could be classified as idiopathic and due to other medical reasons, i.e., secondary CTS. Most instances of CTS are considered to be idiopathic. Other factors, for example, age, hereditary, and anthropometric components, have been implicated in the risk factors of idiopathic CTS [10]. Obesity, diabetes, and hypothyroidism have been associated with a double chance of developing CTS due to increased intraneural pressure in the carpal tunnel or vascular deficits [11].

CTS is usually diagnosed clinically by examining signs and symptoms, which are then assessed by Tinel's test and Phalen's test along with nerve conduction studies and electromyography, which can be valuable for deciding the severity of the median nerve lesion [12]. Scientific literature for the treatment of CTS has given conflicting results. A recent review concluded that surgical management is better compared to splinting for CTS treatment [13]. Butler found that although surgical release has led to a superior outcome than physiotherapy, the clinical significance of this distinction was small. It was also reported in this study that 61% of CTS patients with mild to moderate symptoms preferred physiotherapy treatment to any kind of surgical treatment [14]. Local and oral steroid therapies have shown strong results in the conservative treatment of CTS [15].

Neuromobilization is a manual therapy treatment that alters the physiological properties of nerves, and there is likelihood that its methods especially the sliding technique may have beneficial effects on patients with CTS [6]. Nerve sliding techniques can improve the symptoms when performed at the end of range of motion [16]. Neuromobilization interventions reduce pain in CTS as per literature [17–19]. CTS patients showing lower hyperexcitability respond better to neuromobilization, but still evidence is not obvious according to different studies [20]. Another review has concluded that reported improvements in pressure pain threshold, pain, and function of CTS patients after nerve gliding, combined or not with supplementary therapies, when comparing nerve gliding with other therapies [21].

Neural gliding is a treatment technique that improves the symptoms of CTS. Evidence demonstrates that median nerve excursion can be influenced by neural gliding technique, as shown in a cadaveric study [22]. De-la-Llave-Rincon et al. concluded that the application of soft tissue mobilization and neurodynamic techniques decreased the intensity of pain but did not change pressure pain sensitivity in the group of women with chronic CTS [1].

Going through the literature, there are many treatment options for CTS including conservative and surgical management. However, no one is a better treatment option than another. Therefore, the evidence regarding treatment for the most appropriate strategic option is not clear. Moreover, surgical treatment is very costly as compared to conservative treatment. So, there is a need for more research to use neuromobilization as a better treatment option. Little work has been done with the use of neuromobilization in CTS patients, and no comparative study of neuromobilization with conventional physical therapy treatment, including ultrasonic therapy, splinting, and tendon gliding exercises, has been done so far. This study is aimed at determining benefits of neuromobilization in addition to conventional treatment for CTS. Therefore, this study will be helpful for the treatment of CTS in mild to moderate conditions.

## 2. Materials and Methods

### 2.1. Study Design

This was a prospective, single-blinded randomized clinical controlled trial comparing routine physical therapy with and without neuromobilization in patients with mild to moderate carpal tunnel syndrome. The patients were screened by an independent assessor and randomly allocated into either an experimental group or a control group. Randomization was stratified by another person and severity using randomly permuted blocks of four or six patients. After recruitment, the stratification person was contacted for allocation so that randomization could be secured and concealed.

The participants and treatment-giving therapists were not blinded. The assessor was blinded. All outcomes were being measured by an investigator who was blinded to group allocation.

### 2.2. Participants

A total sample of 66 patients was taken in this study. A sample size was calculated using G∗Power version 3.1.9.3 using the Group 1 mean 2.2, Group 2 mean 2.9, effect size 0.5, alpha error 0.05, power of study 0.8, and allocation ratio which was taken as 1 [11]. They did not report standard deviation, and there was no other article available, so we assumed SD = 1 for both groups. CTS patients aged 20–45 with less than a three-month history of CTS were recruited for the study. Diagnosis and mild to moderate severity of CTS were confirmed using physical tests and electromyography. The participants were excluded if they suffered from any systemic or musculoskeletal pathology of the involved extremity and if they had been suffering from CTS for more than three months, with severe to extreme symptoms, and also confirmed by electromyography, history of any previous surgery or corticosteroid injection treatment for CTS, any sensory or motor deficit in the ulnar or radial nerve, recurrent CTS, and median nerve involvement above the wrist. Individuals were recruited from Mayo Hospital Lahore from August 2019 to June 2020. The intervention was given in the Outdoor Physiotherapy Department of Mayo Hospital Lahore. The University Ethics Committee approved the protocol of the study, and all patients gave their written voluntary informed consent before participation.

### 2.3. Outcome Measures

Objective measures were pain on the numeric pain rating scale (NPRS), range of motion measured by goniometer, and strength using grades of manual muscle testing. Wrist ROM was measured using biaxial goniometers placed on the dorsal side of the right and left wrists, with the proximal part in the midline between the radius and the ulna and the distal part over the third metacarpal bone. Wrist ROMs measured include flexion, extension, radial, and ulnar deviations. MMT was conducted with the therapist's index finger opposing the patients' thumb abduction or index finger abduction. All tests were performed by the same person. MMT was scored on a scale of 0 to 5 based solely on resistance (0–1 no resistance, 2–4 decreased resistance, and 5 normal). The subjective measure was as follows: functional limitation is measured by the Boston Carpal Tunnel Syndrome Questionnaire (BCTQ), which has two subscales: the symptom severity scale (SSS) and the functional status scale (FSS).

### 2.4. Assessment

Patients were recruited from Mayo Hospital Lahore. A qualified assessor examined the patient. Physical assessment was made through reverse Phalen's test and Phalen's and Tinel's tests [23–25]. The diagnosis was confirmed using nerve conduction studies (NCS) with electromyography (EMG). An informed consent form was taken from selected patients. The numeric pain rating scale, manual muscle testing for strength, goniometer for range of motions, and Boston Carpal Tunnel Syndrome Questionnaire for functional limitation were measured.

### 2.5. Intervention

Patients were divided into two groups randomly. Group 1 was the control group and Group 2 was the experimental group. Group 1 received conservative treatment including an ultrasound therapy two days a week for 6 weeks, using a pulsed mode 0.8 W/cm^2^ and frequency 1 MHz [26], wrist splinting, and tendon gliding exercises, while Group 2 received both conservative treatments including ultrasound, splinting, and tendon gliding exercises as well as neuromobilization technique. The neuromobilization technique included passive neuromobilization of the median nerve and functional self-exercises. The neuromobilization procedure started with the patient in the supine position. The following steps were taken in sequence: slight glenohumeral abduction, then shoulder girdle depression, then elbow extension with arm lateral rotation and forearm supination, then wrist, finger, and thumb extension were added, and in the end, the shoulder was taken into further abduction. To apply maximum stretch on the opposite cervical side, flexion was done first, and then, in the end, the wrist was repeatedly moved into and out of stretch by performing a few degrees of flexion and extension at the wrist [27]. All movements were taken to the end of available ROM. Three sets of 15 repetitions of median nerve mobilization were performed during each session.

Patients were treated by the physical therapist for 2 sessions a week for up to 6 weeks. Clinical findings were taken before the first treatment session, after a three-week treatment period, and then after six weeks. Interventions for both groups were given by experienced physiotherapists, as shown in Figure 1.

### 2.6. Data Analysis

For data analysis, IBM SPSS v. 21 was used. Mean ± SD was used for quantitative data and frequency (%) for qualitative data, whereas pp-plot and qq-plot were used along with the one-sample Kolmogorov-Smirnov test to check the normality of data. As the data was normally distributed for comparison of quantitative data in groups, an independent sample *t*-test was applied at each follow-up separately. Multivariate repeated measurement ANOVA was applied to compare quantitative data within and between the groups. *P* value < 0.05 was taken as significant.

## 3. Results

Table 1 shows a pretreatment comparison of characteristics of both groups. There was no significant difference between the groups (*P* > 0.05), and both groups were comparable in their characteristics.

Table 2 represents the frequencies of categorical variables. Figure 1 shows the recruitment strategy and experimental plan for the study. Out of 100 patients referred by the neurologist with confirmed CTS, 25 were suffering from severe signs and symptoms due to which they were excluded from the study. The rest of the 75 patients were counseled about the research and were asked for consent. Out of these 9 patients who did not agree and were dropped out of the study, the remaining 66 patients were randomly divided into two groups and reassessment was done at the end of the 3^rd^ and 4^th^ week. At the end of the third week, there were seven dropouts, five from the routine physical therapy group and two from the neuromobilization group, who were replaced by new participants.

Means and standard deviations of before treatment, at the mid of the treatment, and end of the treatment are shown along with *P* values for with the group change and also for between the group comparisons which are shown in Table 3.

### 3.1. With the Group Comparisons

Repeated measurement ANOVA (Table 3) revealed that variables improved significantly and there was a significant increase in range of motion in all four movements and muscle strength of all four groups, i.e., flexors, extensor, ulna, and radial deviators (<0.001).

Pain measured at NRPS, the severity of symptoms measured by SSS index, activity limitation measured by FSS index, and overall change in symptoms measured by BCTQ also improved statistically with <0.001 shown by repeated measurement ANOVA.

### 3.2. Between the Group Comparisons

An independent sample *t*-test (Table 1) identified that there was not any statistically notable variation between the groups, i.e., the routine physical therapy group and the neuromobilization group, in terms of flexion (0.141), extension (0.06), radial deviation (0.591), ulnar deviation (0.348), flexor strength (0.838), extensor strength (0.703), radial deviator strength (0.461), ulnar deviator strength (0.262), median nerve latencies (0.241), NRPS (0.865), SSS index (0.237), FSS index (0.130), and BCTQ index (0.133). After treatment, an independent sample *t*-test was performed again and *P* values were calculated again, which identified the differences between the groups. There was not any significant difference in muscle strength of all four groups as flexor strength (0.432), extensor strength (0.458), radial deviator strength (0.358), ulnar deviator strength (0.358), and ROM in radial (0.461) and ulnar deviation (0.626). However, after the treatment, flexion (0.05), extension (0.007), pain intensity at NRPS (0.034), symptom severity at SSS index (0.04), FSS (0.017), and BCTQ (0.022) all differed statistically and denoted that the addition of neuromobilization was much better for management of CTS as compared to routine physical therapy.

## 4. Discussion

The results of this research support our hypothesis that the addition of neuromobilization in the rehabilitation program of patients with carpal tunnel syndrome along with routine physical therapy has significant beneficial effects. Although routine physical therapy does improve signs and symptoms significantly, the addition of median nerve mobilization significantly enhances the results. Furthermore, there is no additional benefit of median nerve mobilization in improving muscle strength in patients with CTS.

Although studies have shown that neuromobilization improves pain symptoms and function [16–19], but there are claims that neuromobilization is not a better technique and just routine physical therapy improves symptoms more [28]. That was also supported by a systematic review that describes the effects of neuromobilization in CTS unclear [20]. But our study negates his results and shows that the addition of median nerve mobilization can significantly improve the results of the physiotherapy treatment program. It could be the difference in results is due to different age group as the participants in our study were much younger. In another research that compared exercise in addition to nerve gliding and splinting with ultrasound and splinting and tendon gliding and nerve mobilization, it was found that exercises including tendon gliding along with nerve mobilization and ultrasound had better long-term effects as compared to other techniques [29]. Our results also support these findings, as adding nerve gliding exercises improved results significantly.

Results of Fernandez-De-Las-Penas et al. study in Spain showed that manual therapy is effective in improving pinching and gripping power in CTS patients [30]. One finding of our study was that neuromobilization did not result in a significant increase in muscle strength as compared to other groups. It may be because nerve gliding techniques affect mechanical and physiological properties of the nervous system and improve nerve flow to the muscles and do not directly impact muscles [27]; if a long-term follow-up had been carried out, then changes in muscle strength could have been observed. Also, to measure handgrip strength, we used manual muscle strength testing grades, which are prone to bias because of low interrater and intrarater reliability. Maybe there was a significant change but the assessor could not detect it or mention it as we have five grades for manual muscle testing [31].

In the neuromobilization group, there was a more rapid increase in range of motion and improvement in FSS score as compared to the routine physical therapy group. This may be due to the fact that neuromobilization is usually done at the end of the range of motion by moving the hand into and out of the stretched position. This may result in a rapid increase in range of motion, especially flexion and extension, and hence an increase in functional activities.

In the end, there were some limitations to our study which should be discussed. First of all, the sample size was a convenient sample, which is not a very preferable sampling technique due to the risk of biases. Second, our sample size was small and there was no intention to treat analysis for the dropouts, which could have resulted in a change in results. Third, we used manual muscle testing for muscle strength, which resulted in similar results in both groups. The use of an electronic muscle strength meter could have given better results. The results of this study are short term as we did not follow up the patients after six weeks. In the end, this study was a self-financed study due to which we could not get posttreatment electromyography and nerve conduction studies. This paves the way for studies that are more organized and better funded so that gaps that occurred in our study due to financial and organizational constraints can be filled.

## 5. Conclusion

This study concluded that the addition of neuromobilization in rehabilitation programs of patients with mild to moderate carpal tunnel syndrome can result in better outcomes in terms of range of motion, pain, functional outcomes, and symptom severity. With the addition of neuromobilization, although there was an increase in muscle strength, it was significant when compared with the other groups. The effect of neuromobilization is only short term, and the further effect at midterm or long term is not clear.

## Figures and Tables

**Figure 1:** CONSORT flow diagram.

**Table 1:** Baseline comparison of both groups.

	Routine physical therapy group	Neuromobilization group	*P* values
	Mean ± Std.dev.	Mean ± Std.dev.	
Age of the participant	37.79 ± 5.91	35.58 ± 7.15	0.327
Weight of the patient	69.22 ± 8.62	68.54 ± 9.63	0.741
Height (m)	1.580 ± 0.06	1.62 ± 0.06	0.065
BMI	27.74 ± 4.18	26.20 ± 4.53	0.618
Active wrist flexion of the involved side	47.39 ± 7.77	49.97 ± 6.17	0.141
Active wrist extension of the involved side	47.09 ± 8.27	50.48 ± 5.91	0.06
Active radial deviation of the involved side	12.52 ± 4.22	12.00 ± 3.50	0.591
Active wrist ulnar deviation of the involved side	16.30 ± 5.48	15.18 ± 4.05	0.348
Flexor strength of the involved side	3.15 ± 0.67	3.18 ± 0.52	0.838
Extensor strength of the involved side	3.12 ± 0.74	3.18 ± 0.52	0.703
Radial deviation strength of the involved side	3.09 ± 0.76	3.21 ± 0.54	0.461
Ulnar deviation strength of the involved side	3.09 ± 0.72	3.27 ± 0.57	0.262
Intensity of pain at NPRS	7.33 ± 1.55	7.39 ± 1.32	0.241
Median nerve distal latency (ms)	4.56 ± 0.89	4.32 ± 0.74	0.865
SSS index	2.70 ± 0.58	2.55 ± 0.41	0.237
FSS index	2.83 ± 0.64	2.59 ± 0.64	0.130
BCTQ	5.54 ± 1.13	5.15 ± 0.94	0.133

BMI: body mass index; SSS: symptom severity scale; FSS: functional status scale; BCTQ: Boston Carpal Tunnel Syndrome Questionnaire.

**Table 2:** Characteristics of patients who participated in this study.

	Routine physical therapy group	Neuromobilization group
Gender		
Male	3 (9.1%)	2 (6.1%)
Female	30 (90.9)	31 (93.9%)
Marital status		
Married	29 (87.9%)	24 (72.7%)
Single	4 (12.1%)	9 (27.3%)
Socioeconomic status		
Upper class income above 50000 pkr	8 (24.2%)	10 (30.3%)
Middle class income between 20000 to 50000 pkr	20 (60.6%)	20 (60.6%)
Lower income class income below 20000 pkr	5 (15.2%)	3 (9.1%)
Occupation		
Sedentary worker	12 (36.4%)	5 (15.2%)
Laborer	2 (6.1%)	3 (9.1%)
Housewife	16 (48.5%)	20 (60.6%)
Any other	3 (9.1%)	5 (15.2%)
Effected side		
Right	16 (48.5%)	21 (63.6%)
Left	17 (51.5%)	12 (36.4%)
Vigorous activity		
Yes	10 (30.3%)	8 (24.2%)
No	23 (69.7%)	25 (75.8%)

**Table 3:** Inter- and intragroup comparison between routine physical therapy and neuromobilization groups for the selected parameters after 6 weeks of intervention.

	Routine physical therapy group				Neuromobilization group				*P* value for between the group difference
	Pretreatment	After 3rd week	After 6 weeks	*P* value	Pretreatment	After 3rd week	After 6 weeks	*P* value	
	Mean ± Std.dev.	Mean ± Std.dev.	Mean ± Std.dev.		Mean ± Std.dev.	Mean ± Std.dev.	Mean ± Std.dev.		
Flexion	47.39 ± 7.77	53.67 ± 7.27	61.00 ± 6.76	<0.001	49.97 ± 6.17	57.48 ± 4.94	63.70 ± 4.22	<0.001	0.05
Extension	47.09 ± 8.27	53.94 ± 6.991	53.94 ± 6.99	<0.001	50.48 ± 5.91	50.48 ± 5.91	50.48 ± 5.91	<0.001	0.007
Radial dev.	12.52 ± 4.22	14.70 ± 4.44	14.70 ± 4.44	<0.001	12.00 ± 3.50	12.00 ± 3.50	12.00 ± 3.50	<0.001	0.461
Ulnar dev.	16.30 ± 5.48	20.03 ± 5.31	20.03 ± 5.31	<0.001	15.18 ± 4.05	15.18 ± 4.05	15.18 ± 4.05	<0.001	0.626
Flexor strength	3.15 ± 0.66	3.79 ± 0.69	4.21 ± 0.65	<0.001	3.18 ± 0.52	4.00 ± 0.50	4.33 ± 0.59	<0.001	0.432
Extensor strength	3.12 ± 0.74	3.76 ± 0.70	4.18 ± 0.72	<0.001	3.18 ± 0.52	3.97 ± 0.52	4.30 ± 0.58	<0.001	0.458
Radial dev. strength	3.09 ± 0.76	3.76 ± 0.70	4.18 ± 0.72	<0.001	3.21 ± 0.54	4.03 ± 0.52	4.33 ± 0.59	<0.001	0.358
Ulnar dev. strength	3.09 ± 0.72	3.76 ± 0.70	4.18 ± 0.72	<0.001	3.27 ± 0.57	4.00 ± 0.50	4.33 ± 0.59	<0.001	0.358
Pain at NPRS	7.33 ± 1.55	4.94 ± 1.3	2.73 ± 1.54	<0.001	7.39 ± 1.32	4.48 ± 1.09	1.97 ± 1.28	<0.001	0.034
SSS index	2.70 ± 0.58	1.72 ± 0.60	0.99 ± 0.66	<0.001	2.55 ± 0.41	1.56 ± 0.40	0.73 ± 0.33	<0.001	0.048
FSS index	2.83 ± 0.64	2.18 ± 1.96	1.04 ± 0.58	<0.001	2.59 ± 0.64	1.49 ± 0.42	0.75 ± 0.35	<0.001	0.017
BCTQ index	5.54 ± 1.13	3.91 ± 2.07	2.03 ± 1.19	<0.001	5.15 ± 0.94	3.05 ± 0.69	1.48 ± 0.60	<0.001	0.022

BMI: body mass index; SSS: symptom severity scale; FSS: functional status scale; BCTQ: Boston Carpal Tunnel Syndrome Questionnaire; Dev.: deviation.

## Data Availability

Data will be available on request through an online repository.
